# Inhibition of DNAJC12 Inhibited Tumorigenesis of Rectal Cancer via Downregulating HSPA4 Expression

This article has been retracted.

**DOI:** 10.1155/2022/1027895

**Published:** 2022-09-21

**Authors:** Qi Sun, Yan Lv, Weihua Sun

**Affiliations:** ^1^Third Ward of Cancer Center, The PLA Navy Anqing Hospital, Anqing 246003, Anhui, China; ^2^Department of Oncology, Qingdao Municipal Hospital, Qingdao 266071, Shandong, China

## Abstract

**Background:**

Dysregulation of DnaJ heat shock protein family (HSP40) member C12 (DNAJC12) is implicated in the malignancy progression of multiple cancers. The current study aimed to determine the biology function and mechanism of DNAJC12 in rectal cancer (RC).

**Methods:**

RC tissues, adjacent tissues, RC cell lines, and normal colorectal epithelial cell lines were collected to analyze DNAJC12 expression. The abilities of DNAJC12 on proliferation, migration, and apoptosis of RC cells were detected by CCK-8, wound healing, and flow cytometry assays. Co-IP assays were carried out to confirm the association between DNAJC12 and HSPA4. The effect of DNAJC12 on tumor growth was detected by using the xenograft model of nude mice.

**Results:**

Elevation of DNAJC12 was uncovered in RC tissues and cell lines. DNAJC12 upregulation facilitated RC cell proliferation and migration and induced apoptosis, while DNAJC12 interference showed the opposite results. Besides, HSAP4 served as a potential binding protein for DNAJC12. Rescue experiments revealed that elevated of HSAP4 restored the impact of DNAJC12 silencing on the cell functions. Finally, DNAJC12 silencing hampered tumor growth of RC in vivo.

**Conclusion:**

In summary, this study highlighted a key player of DNAJC12 in modulating the malignant biological progression of RC via DNAJC12/HSPA4 axis, displaying a potential therapeutic target for RC.

## 1. Introduction

Rectal cancer (RC) is one of the most common malignancies of the digestive tract, accounting for approximately more than 30% of colorectal cancer cases [1]. It occurs between the junction of the sigmoid colon and rectum to the dentate line, in a position deep to the pelvic cavity. The incidence of RC has been increasing in frequency over recent years, with nearly 700,000 deaths annually, and the diseased population is becoming younger and younger [2]. At present, the treatment of early RC is mainly surgery, and middle and advanced rectal cancer is mostly treated with radiotherapy and chemotherapy [3]. Patients with advanced RC often have a worse prognosis than patients in the early stage due to the deterioration of their condition, tumor cells undergo metastasis and invasion, which seriously affect the physical health and life safety of patients [4]. Investigations have shown that RC is associated with diet, lifestyle, and genetic heritability in the population, but the specific pathogenesis remains unknown [5, 6]. Therefore, it is beneficial for the prevention and treatment of rectal cancer to study the related factors affecting the occurrence and development of RC from the molecular level and find new therapeutic targets.

DnaJ heat shock protein family (HSP40) member C12 (DNAJC12) is a member of heat shock proteins (HSPs) family that functions as a molecular chaperone to regulate protein folding, processing, maturation, and gene expression [7, 8]. Besides, DNAJC12, also known as JDP1 or HPANBH4, is a protein containing J domain, which is involved in the occurrence and development of many diseases. Accumulated literature indicated that DNAJC12 mutations are associated with nonprogressive Parkinson's disease [7, 9]. Cumulative evidence has suggested that the DNAJC12 variant has been found in patients with mild hyperphenylalaninemia, and it is also a new cause of hereditary hyperphenylalaninemia (HPA) [10, 11]. And, development of dystonia and intellectual disability in humans is strongly associated with biallelic mutations in the DNAJC12 gene [12]. In recent years, many literature studies have reported that the biological role of DNAJC12 has been gradually found in cancer progression, such as gastric cancer, breast cancer, and lung cancer, and DNAJC12 was involved in cancer cell proliferation, migration, invasion, and drug resistance [13–15]. Targeting DNAJC12 in the treatment of RC is still on the way, there are many mechanisms and problems that need to be further explored.

In this work, we proved that DNAJC12 acts as an oncogene in RC progression by binding with HSPA4. Our results may provide relevant information for the research, diagnosis, treatment, and development of related targeted agents for RC.

## 2. Materials and Methods

### 2.1. Source of Tissue Specimens

The RC tissue specimens of all study subjects used in the experiments were derived from patients who underwent curative resection for RC between 2015 and 2020 at the Qingdao Municipal Hospital, a total of 55 cases. All collected tissues were immediately preserved in liquid nitrogen for subsequent experiments. Tissue samples were used in strict compliance with regulations related to human tissue samples from Qingdao Municipal Hospital. Informed consent was obtained from all patients before the study.

### 2.2. Cell Culture

Human RC cell lines (SW1463, SW873, and SW480) and normal human colorectal epithelial cell line (FHC) were provided by the Chinese Academy of Sciences (Shanghai, China). 10% FBS was added into DMEM and then incubated with the above cells in a 5% CO_2_ incubator at 37°C.

### 2.3. Cell Transfection

GeneChem company (Shanghai, China) provided overexpression plasmid of DNAJC12 and HSPA4 shRNA targeting DNAJC12 (sh-DNAJC12: 5′-GGATGTGATGAACTATCTT-3′) and above corresponding negative controls (sh-NC: 5′-TTCTCCGAACGTGTCACGT-3′). SW480 cells were transfected with pcDNA-3.1, DNAJC12, sh-NC, or sh-DNAJC12 by utilizing Lipofectamine 3000 when the cells were approximately 70% confluent. Briefly, an Opti-MEM medium was added to Lipofectamine 3000, and mixed well. At the same time, the Opti-MEM medium and p3000™ reagent were sequentially added to the above DNA plasmids to prepare the DNA master mix. Then, in each test tube, dilute DNA and diluted Lipofectamine 3000 were mixed in proportion (1 : 1). Finally, DNA-liposome complexes were added to the cells after 5 min incubation at room temperature.

### 2.4. Cell Viability Assay

SW480 cells were gradient inoculated in 96-well plates *s* (2.5 × 10^3^/well), followed by 10 *μ*L of CCK-8 solution to 100 *μ*L of cell culture medium, incubated at 37°C for 1 h, and the absorbance of A450 was determined by a microplate reader.

### 2.5. Wound-Healing Assay

Several straight lines were marked across the six-hole plate on the back of the six-hole plate with a marker and ruler, and the spacing of each two straight lines was 0.5 cm. SW480 cell suspension was inoculated into 6-well plates, and the number of cells in each well was 6 × 10^5^. The cells were covered overnight, and the culture medium was discarded. The 10 *µ*L sterile spear head was used to mark the line evenly and slowly perpendicular to the back of the six-hole plate. Cells were gently rinsed with PBS twice to remove the suspended cells. 2 mL of the serum-free medium was added to each well and photos were taken under an inverted microscope. The cells were further cultured and photographed at 24 hours to observe the migration of cells in each well. Image J software was used to measure the area of the scratch area.

### 2.6. Cell Cycle Assay

The cell cycle was checked using the cell cycle staining kit (MultiSciences Biotech Ltd., China). Briefly, SW480 cells were cultured and the number of cells in each well was 5 × 10^5^. After being fixed in 70% ethanol overnight, SW480 cells were gently rinsed with PBS, and further stained with PI for 30 min and stored in darkness. Finally, the cells ratio in different phases was measured using flow cytometry.

### 2.7. Cell Apoptosis Assay

For cell apoptosis analysis, Annexin V-PI apoptosis detection kit I (BA1250, EnoGene, China) was performed. First, SW480 cells were collected and 500 *μ*L of binding buffer resuspend cells. After Annexin V-FITC was added to the mixture, PI was added to the mixture again and incubated for 10 min in the dark at room temperature. Using flow cytometry, the cell staining and cell apoptosis ratio was analyzed.

### 2.8. Coimmunoprecipitation (CoIP) Assay

SW480 cells are lysed in lysis buffer to obtain cell lysate, followed by being incubated with agarose bead-conjugated antibodies against anti-DNAJC12 and anti-HSPA4 (1 : 1500) overnight. Subsequently, the beads were washed to harvest the binding proteins. Finally, the western blotting was used to assess immunoprecipitated protein.

### 2.9. Western Blot Assay

Sample cells or tissue culture dishes were placed on ice and RIPA-containing cell lysate was added, followed by determination of protein content. The equal amount of protein (20 *μ*g) and the 10% concentration SDS-PAGE gel was configured for electrophoresis. After completion of electrophoresis, a methanol-activated PVDF membrane was used for protein transfer. Next, primary antibodies against DNAJC12, HSPA4, and GAPDH were used to incubate with the membrane overnight after blocking with 5% fat-free milk and HRP-conjugated secondary antibodies were further used to incubate with the membrane for 2 h at room temperature. Finally, the ECL working solution was incubated with PVDF membranes for 10–30 s and immediately placed into the ECL imager to visualize protein bands.

### 2.10. Animal Experiments

BALB/c nude mice (male, four-week-old) were raised in the animal experiment center of Qingdao University and reserved in our hospital with the approval of the ethics committee of our hospital. For establishing nude mice RC subcutaneous transplanted tumor model, table transfected cell lines SW480/sh-NC and SW480/sh-DNAJC12 were cultured, respectively. Then, the SW480 transfected cells (1 × 10^6^) were inoculated subcutaneously in mice. The mice were observed for four weeks, and then euthanatized through intraperitoneally anesthetizing with 1% pentobarbital sodium (100 mg/kg) to remove the tumors. Tumor sizes were determined by Vernier caliper measurements, and tumor volumes were calculated according to the formula: ((shortest diameter)^2^ × (longest diameter))/2.

### 2.11. Statistical Analysis

All in vitro and in vivo experiments were repeated more than three times, and the results were expressed as mean ± standard deviation. Moreover, the Shapiro–Wilk test was utilized to verify that the data were normally distributed. The Levene test was utilized to verify the homogeneity of variances. Next, the differences between the two groups were compared by Student's *t*-test, while between multiple groups compared by one-way analysis of variance (ANOVA). The Kruskal–Wallis test followed by the post hoc analysis (Mann–Whitney *U* test) was utilized to assess pairwise differences among the adjusted means. Statistical calculations were performed using SPSS 22.0 software, where a *p* value < 0.05 indicates a significant difference.

## 3. Results

### 3.1. DNAJC12 Was Upregulated in RC Tissues and Cell Lines

In order to investigate whether there is a link between the expression of DNAJC12 and the development of RC, we first assessed DNAJC12 level in RC tissues and adjacent tissues, and uncovered that DNAJC12 in RC tissues was remarkably higher than that in adjacent tissues (Figure 1(a)). Subsequently, we found that patients with a high level of DNAJC12 was substantially associated with shorter overall survival through Kaplan–Meier survival curve (Figure 1(b)). Furthermore, analysis of GEPIA database showed that DNAJC12 was differentially expressed in TNM stages I, II, III, and IV. Among them, there was significant difference among the four groups (Figure 1(c)). To further confirm the results of the above analysis, we examined the expression of DNAJC12 in RC cell lines. As expected, the results of western blotting showed that DNAJC12 was elevated in RC cell lines (SW1463, SW837, and SW480) compared with normal human colorectal epithelial cell line (FHC) (Figure 1(d)).

### 3.2. DNAJC12 Regulated Cell Proliferation, Migration, and Apoptosis in RC

In order to further explore the biological function of DNAJC12 in RC cells, SW480 cells were transfected with DNAJC12 overexpression plasmid or DNAJC12 shRNA (sh-DNAJC12). Western blotting results showed that transfection with DNAJC12 exhibited a better upregulating capacity and transfection with sh-DNAJC12 which exhibited a better silencing capacity compared with their negative control, respectively (Figure 2(a)). CCK8 results uncovered that upregulation of DNAJC12 prominently improved cell proliferation in SW480 cells, while silencing of DNAJC12 had the opposite effect (Figure 2(b)). Using flow cytometry, we indicated that upregulation of DNAJC12 expression significantly accumulated S phase and suppressed G0/G1 cycle arrest of SW480 cells, thus contributing to cell proliferation (Figure 2(c)). Conversely, DNAJC12 silencing exerted an opposite effect in SW480 cells (Figure 2(c)). Wound-healing assays demonstrated that DNAJC12 elevation effectively promoted the migration of SW480 cells, while DNAJC12 silencing prominently reduced the migration of SW480 cells (Figure 2(d)). Besides, upregulation of DNAJC12 effectively reduced the percentage of apoptotic cells, while interference of DNAJC12 showed opposite results (Figure 2(e)).

### 3.3. DNAJC12 Interacted with HSPA4

Next, we further examined the potential biological mechanism of DNAJC12 in RC progression. Using the STRING database, we found that HSPA4 was a potential downstream protein of DNAJC12 (Figure 3(a)). In addition, the results of GEPIA database analysis indicated that HSPA4 expression level in RC patients (*n* = 92) was remarkably higher than in heathy humans (*n* = 318) (Figure 3(b)). Western blotting assays demonstrated that compared to the normal adjacent tissues, RC tissues displayed increased expression of DNAJC12 (Figure 3(c)). And, we also observed that DNAJC12 level was overexpressed in SW1463, SW837, and SW480 compared with FHC (Figure 3(d)). Through correlation analysis, we suggested that expression of HSPA4 was positively correlated with DNAJC12 in RC tissues (Figure 3(e)). Furthermore, the results of CoIP assays uncovered that HSAP4 existed in complexes precipitated with antibody against DNAJC12 compared with control IgG (Figure 3(f)).

### 3.4. DNAJC12 Played a Carcinogenic Role by Regulating HSPA4 Expression

To explore whether HSPA4 was involved in DNAJC12-mediated biological function in RC development, we performed the rescue assays. Surprisingly, the results of western blotting demonstrated that transfection with sh-DNAJC12 efficiently reduced HSPA4 expression, which was restored by transfection with HSPA4 (Figure 4(a)). Then, CCK-8 assay demonstrated that HSPA4 overexpression significantly abolished the DNAJC12-mediated inhibitory effect on cell proliferation (Figure 4(b)). HSPA4 upregulation reversed DNAJC12 silencing-induced the G0/G1 arrest by (Figure 4(c)). The results of wound-healing and flow cytometry assays demonstrated that DNAJC12 interference suppressed migration and accelerated apoptosis of SW480 cells, whereas HSPA4 overexpression could invert these changes (Figures 4(d) and 4(e)).

### 3.5. DNAJC12 Knockdown Repressed Tumor Growth of RC

To further explore the influence of DNAJC12 in RC, a subcutaneous tumor model of RC mice was established in nude mice. After 4 weeks, we uncovered that tumor growth was effectively restrained in the DNAJC12 silencing group compared to the sh-NC group, as indicated by a significant reduction in tumor volume and weight (Figures 5(a)–5(c)). In addition, compared with the sh-NC group, we further found that DNAJC12 was remarkably reduced in the sh-DNAJA12 group (Figure 5(d)). Also, HSPA4 protein level was found to dramatically reduce in the sh-DNAJA12 group (Figures 5(e) and 5(f)).

## 4. Discussion

Rectal cancer (RC) is one of the malignant tumors with high incidence rate and mortality. It is easy to relapse after treatment, causing a major threat to the health and life safety of patients [16, 17]. With the development of biotechnology, searching for therapeutic targets and prognostic predictors in patients with RC at the molecular level has become a research hotspot. DNAJC12 has many biological functions and plays an important role in tumor diseases. For example, the level of DNAJC12 mRNA in gastric cancer was substantially higher than that in normal adjacent tissues, and upregulation of DNAJC12 in gastric cancer resulted in remarkably shorter overall survival of gastric cancer patients and also was closely related to the invasive phenotype of gastric cancer [13]. A previous study revealed that DNAJC12 was an estrogen target gene, and high levels of DNAJC12 were found in MCF-7 breast cancer cells after 17beta-estradiol treatment [14]. In lung cancer, DNAJC12 silencing memorably suppressed lung cancer cell growth, as indicted by a significant reduction in proliferation, colony formation, migration, and invasion and increase in cell apoptosis by modulating *β*-catenin expression and activation [15]. Besides, HNF1A enhanced the expression of DNAJC12 in nonsmall cell lung cancer by promoting the transcription of DNAJC12, thus promoting aerobic glycolysis and resistance development of DDP through regulating *β*-catenin expression [18]. However, there are few reports on DNAJC12 in RC. He et al. demonstrated that overexpression of DNAJC12 in RC tissues has been found, and the degree of expression correlates with poor prognosis, such as overall survival, disease-free survival, and local recurrence-free survival [19]. Therefore, it is necessary to study the role and potential mechanism of DNAJC12 in the occurrence and development of RC. Here, in consistence with previous literature studies, we uncovered that DNAJC12 is overexpressed in RC tissues and cell lines. Upregulation of DNAJC12 was statistically correlated with TNM stages and reduced survival rate in RC. Additionally, we showed that DNAJC12 promoted RC progression by mediating proliferation, migration, and apoptosis of RC cells.

Heat shock 70 kDa protein 4 (HSPA4) is a member of HSP110 family, which plays an important role in inflammation, human immunity, and tumor [20]. In Parkinson's disease, HSPA4 inhibited neuroinflammation through deacetylation with SIRT1, which lead to neuroprotection [21]. HSPA4 has been found to regulate the immune response in the gut, which alleviated the symptoms of gastric ulcer by restraining SDF-1 and twist expression in fibroblasts [22]. Of note, HSPA4 has been demonstrated to be elevated in tissues from hepatocellular carcinoma patients and head and neck squamous cell carcinoma patients, and associated with poor overall survival [23, 24]. It was also reported that HSPA4 was involved in proliferation, differentiation, and metastasis of tumor cells. Nan et al. demonstrated that HSPA4 elevated accelerated endoplasmic reticulum stress, cell growth, triple-negative breast cancer cell migration, and invasion abilities by activating the Syntenin/SOX4/Wnt/*β*-catenin pathway [25]. Intriguingly, current evidence shows that HSPA4 plays an important role in intestinal diseases [26, 27]. And, high level of HSPA4 was uncovered to be elevated in colorectal cancer tissues, and downregulation of HSPA4 reduced proliferation and migration, induced G2-phase cycle arrest and apoptosis of colorectal cancer cells as well as suppressed xenograft growth though inactivating the PI3K/AKT pathway [28]. Wang et al. revealed that high levels of HSPA4 in patients with RC predicted poor response to neoadjuvant concurrent chemoradiotherapy [29]. In our research, we provided the first evidence of the binding between DNAJC12 and HSPA4 in RC. Besides, rescue assay showed that HSPA4 overexpression reversed the inhibitory effect of DNAJC12 interference on the malignant progression of RC cells.

In conclusion, our study identified that DNAJC12 was upregulated in RC tissues and cells. DNAJC12 elevated contributed to HSPA4 expression and ultimately accelerated the malignant progression of RC. This study provided a new insight into the regulatory mechanisms of DNAJC12 on RC progression.

## Figures and Tables

**Figure 1:** DNAJC12 was overexpressed in RC tissues and cell lines. (a) Western blotting was used to analyze the relative expression of DNAJC12 in RC tumor tissues (*n* = 55) and adjacent tissues (*n* = 55). (b) Influence of DNAJC12 on RC overall survival. (c) GEPIA database was used to analyze the relative expression of DNAJC12 at TNM stages I II, III, and IV. (d) Western blotting was used to analyze the relative expression of DNAJC12 in RC cell lines SW1463, SW837, and SW480, and normal human colorectal epithelial cell line (FHC). ^*∗*^*P* < 0.05.

**Figure 2:** DNAJC12 exerted an oncogene effect by modulating the functional characteristics of RC cells. (a) Western blotting detection of DNAJC12 level in SW480 cells after transfection. (b) CCK-8 detection of SW480 cell proliferation after transfection. (c) Flow cytometry detection of SW480 cell cycle after transfection. (d) Wound-healing detection of SW480 cell migration after transfection. (e) Flow cytometry detection of SW480 cell apoptosis after transfection. ^*∗*^*P* < 0.05.

**Figure 3:** DNAJC12 bound with HSPA4. (a) STRING detection of the relationship of DNAJC12 and HSPA4. (b) GEPIA database analysis of HSPA4 level. (c) Western blotting detection of HSPA4 level in tumor tissues and adjacent tissues (*n* = 55) collected from RC patients. (d) Western blotting detection of HSPA4 level in RC cell lines and FHC cells. (e) Correlation analysis between DNAJC12 and HSPA4. (f) Co-IP validation of the relationship of DNAJC12 and HSPA4. ^*∗*^*P* < 0.05.

**Figure 4:** HSPA4 elevation abolished the impact of DNAJC12 interference in RC cells. (a) Western blotting detection of HSPA4 level in SW480 cells after transfection. (b) CCK-8 detection of SW480 cell proliferation after transfection. (c) Flow cytometry detection of SW480 cell cycle after transfection. (d) Wound-healing detection of SW480 cell migration after transfection. (e) Flow cytometry detection of SW480 cell apoptosis after transfection. ^*∗*^*P* < 0.05.

**Figure 5:** DNAJC12 silencing repressed tumor formation in vivo. Mice subcutaneous xenografts were constructed by injection SW480 cells, transfection with sh-DNAJC12, or sh-NC. (a) Observation of tumor growth following DNAJC12 silencing. (b) Detection of mouse tumor volume following DNAJC12 silencing. (c) Detection of mouse tumor weight following DNAJC12 silencing. (d, e) Western blotting detection of DNAJC12 and HSPA4 level following DNAJC12 silencing. ^*∗*^*P* < 0.05.

## Data Availability

The labeled dataset used to support the findings of this study are available from the corresponding author upon request.
